The article "DDP-resistant ovarian cancer cells-derived exosomal microRNA-30a-5p reduces the resistance of ovarian cancer cells to DDP" was retracted in 2021. Reasons: signs of a paper mill; original data or images not available; concerns about the data; concerns about the images.

# DDP-resistant ovarian cancer cells-derived exosomal microRNA-30a-5p reduces the resistance of ovarian cancer cells to DDP

**DOI:** 10.1098/rsob.190173

**Published:** 2020-04-29

**Authors:** Ronghua Liu, Yucan Zhang, Peiwen Sun, Changxiu Wang

**Affiliations:** 1 Department of Obstetrics, Linyi People's Hospital, Linyi 276000, People's Republic of China; 2 Department of Surgery, People's Hospital of Luozhuang District, Linyi 276000, People's Republic of China

**Keywords:** ovarian cancer, exosomes, microRNA-30a-5p, SRY-box 9, DDP, drug resistance

## Abstract

Exosomes carrying microRNAs (miRNAs) have been demonstrated to play critical roles in the regulation of development, growth and metastasis of cancer. Bioinformatic predictions identified differentially expressed SRY-box 9 (SOX9) in OC, and the regulatory miRNA miR-139-5p. Here, we aim to evaluate the function of exosomal miR-139-5p in the sensitivity of ovarian cancer (OC) cells to cis-diamminedichloroplatinum(II) (DDP). Expression pattern of miR-139-5p and SOX9 in ovarian cancer cells (SKOV3) and DDP-resistant cells (SKOV3/DDP) was identified using reverse transcription quantitative polymerase chain reaction and western blot analysis. The relationship between miR-139-5p and SOX9 was validated using a dual-luciferase reporter assay. SKOV3/DDP cell line was developed and introduced with miR-30a-5p mimic to analyse the effects of miR-30a-5p on resistance to DDP. The *in vitro* and *in vivo* effects of exosomal miR-30a-5p on resistance of SKOV3 cells to DDP were assessed in a co-culture system of exosomes and OC cells as well as in tumour-bearing nude mice. High expression of SOX9 and low expression of miR-30-5p were witnessed in OC. Furthermore, miR-30-5p, a downregulated miRNA in SKOV3/DDP cells, increased the rate of cell apoptosis and enhanced the sensitivity of SKOV3/DDP cells to DDP by targeting SOX9. Moreover, exosomes carrying miR-30a-5p were identified to sensitize SKOV3/DDP cells to DDP both *in vitro* and *in vivo*. These data together supported an important conclusion that DDP-resistant OC cell-derived exosomal miR-30a-5p enhanced cellular sensitivity to DDP, highlighting a potential strategy to overcome drug resistance.

## 1. Introduction

Ovarian cancer (OC) is one of the most life-threatening gynaecological malignancies for women globally. It ranks seventh among common cancers in female population and eighth among cancer-related deaths overall, with 5-year survival rates below 45% [1]. Contemporary treatment of OC involves aggressive tumour cytoreductive surgery followed by platinum-based multiagent chemotherapy [2]. However, the resistance of tumour cells to chemotherapy or molecular-targeted therapies limits the effectiveness of current cancer therapies [3]. Despite cis-diamminedichloroplatinum(II) (DDP) having been widely applied as an effective chemotherapeutic drug to treat OC alone and in combination with other therapeutic methods [4], emerging resistance to DDP is a current challenge in the therapy of OC [5]. Despite the liposomal application of DDP in current clinical cases, there are few reports about approaches for overcoming DDP resistance [6]. Therefore, it is urgent to develop novel strategies to thwart DDP resistance in OC.

MicroRNAs (miRNAs) are a class of diverse small non-coding RNAs that are able to inhibit the translation and stability of mRNAs, and regulate functional mRNAs involved in key cellular processes such as cell differentiation, migration and apoptosis [7]. The deregulation of miRNAs in disease conditions can be harnessed as potential therapeutics by either miRNA replacement therapy using miRNA mimics or inhibition of miRNA function using anti-miRNAs [8]. In the context of OC, previous work has identified several differentially expressed miRNAs in OC that can serve as diagnostic and prognostic targets for cancer treatment [9], including many that have been specifically implicated in influencing DDP resistance via various mechanisms [10]. For example, a recent study identified an inhibitory effect of miR-30a-5p upon DDP resistance in OC [11]. Apart from the aforementioned miRNA mimic, upregulation of miR-30a-5p in OC cells necessitates more alternative approaches.

Recently, it has been demonstrated that the transfer of miRNAs from omental adipocytes and fibroblasts via micro-vesicles to tumour cells is a promising way to break chemoresistance [12]. Exosomes are saucer-shaped vesicles of 40–150 nm in diameter separated by a lipid bilayer, secreted by various cells [13]. Exosomes are involved in the developmental processes of cancer, affecting the drug resistance, and thus bear potential clinically to be applied as biomarkers, therapeutic targets or engineered nanocarriers [14].

A recent study revealed an association between high SOX9 expression and primary chemoresistance [15]. Intriguingly, miR-30a-5p was predicted to target SOX9 based on the results from a miRNA-target prediction website. Thus, we reasoned that miR-30a-5p might enhance sensitivity to DDP in OC by targeting SOX9. The aim of our study, therefore, is to identify the modulatory effect of exosomal miR-30a-5p on the sensitivity of the OC to DDP with the ultimate goal to find a possible target to overcome drug resistance in OC.

## 2. Result

### 2.1. SOX9 is an upregulated gene in OC

To identify potential OC-associated genes, we analysed three publicly available datasets GSE18520, GSE4122 and GSE54388 using the R software package. For each dataset, we computed the top 200 differentially expressed genes (DEGs) in OC and identified nine candidate genes which were found across all three datasets. These genes were ABCA8, DIRAS3, SOX9, TCF21, PDGFD, CD24, CLDN3, SOX17 and EPCAM (figure 1*a*). We also retrieved the top 20 OC-associated genes from Disease Gene Search Engine with Evidence Sentences (DiGSeE) and these were BRCA1, TP53, PLOD1, MUC16, BRCA2, VEGFA, ERBB2, FSHR, AKT1, SHBG, ESR1, EGFR, MAPK1, BCL2, IGF1, GNRH1, IL6, TNF, ABCB1 and CGA. We then constructed an interaction network of known OC-associated genes and our identified DEGs in the String database (figure 1*b*). Our interaction network suggested that that SOX9 was one of the most relevant candidate genes, and thereby led us to explore its potential role in OC. We summarized the expression of the top 30 DEGs in the GSE4122 as a heatmap in figure 1*c*, and additionally, the expression of SOX9 in GSE18520 and GSE54388 in figure 1*d*,*e*. Overall, through the above unbiased analyses, we identified SOX9 as one of the most upregulated genes in OC tissues compared with normal tissues.

**Figure 1.** SOX9 is highly expressed in OC. (*a*) Intersections of top 200 DEGs in OC among GSE18520, GSE4122 and GSE54388. (*b*) Interaction network of top 20 OC-associated genes and nine DEGs, diamond referring to DEGs and circle referring to OC-associated genes. (*c*) The heatmap illustrating the expression of the top 30 DEGs in the GSE4122, the *x*-axis indicating the sample number, the *y*-axis referring to DEGs, the histogram at the upper right referring to the colour gradation, each rectangle in the figure referring to one sample expression value. (*d*,*e*) The expression of SOX9 in OC in GSE18520 and GSE54388.

### 2.2. miR-30a-5p targets SOX9 in OC

Having discovered SOX9 as a candidate gene upregulated in OC, we used the online prediction tools DIANA, TargetScan, miRDB, miRpath and mirDIP to predict putative miRNAs that regulate SOX9. We summarized our predictions from all four online tools as a Venn diagram (figure 2*a*) and identified one miRNA, miR-30a-5p, which was consistently predicted across all databases. We therefore focused on drilling down on miR-30a-5p given its likelihood in regulating SOX9.

**Figure 2.** miR-30a-5p specifically targets SOX9. (*a*) The miRNAs regulating SOX9 predicted from DIANA, TargetScan, miRDB, miRpath and miRDIP. (*b*) Binding sites between miR-30a-5p and the 3′UTR of SOX9 mRNA and luciferase activity of SOX9-WT and SOX9-MUT after miR-30a-5p mimic transfection. (*c*) The mRNA expression of SOX9 after the overexpression of miR-30a-5p determined by RT-qPCR. (*d*) The protein expression of SOX9 normalized to GAPDH after overexpression or inhibition of miR-30a-5p measured by western blot analysis. *p < 0.05 versus the NC mimic or NC inhibitor group. Measurement data were expressed as mean ± standard deviation. Comparison between two groups was analysed by unpaired *t*-test. Data at different time points were compared by repeated-measures ANOVA, followed by Tukey's *post hoc* test. Cell experiment was repeated three times independently.

In addition to the prediction that miR-30a-5p targets SOX9, the microRNA.org online tool also provided putative binding sites between miR-30a-5p and SOX9. To validate this predicted binding interaction, we constructed a mutation in the binding site and used a dual-luciferase reporter gene assay as the readout (figure 2*b*). While the luciferase activity of the SOX9-Wt in the cells transfected with miR-30a-5p mimic was decreased (*p* < 0.05), the luciferase activity of SOX9-MUT remained unchanged after miR-30a-5p mimic transfection (*p* > 0.05; figure 2*b*), thereby indicating that miR-30a-5p can specifically bind to SOX9. As further validation, we both overexpressed and inhibited miR-30a-5p, and queried SOX9 expression by reverse transcription quantitative polymerase chain reaction (RT-qPCR) and western blot analysis. miR-30a-5p overexpression resulted in a concomitant decrease in both SOX9 mRNA and protein levels, while its inhibition led to an increase in both SOX9 mRNA and protein levels (figure 2*c*,*d*). In summary, the above set of experiments showcase that miR-30a-5p can target SOX9 and downregulate its expression.

### 2.3. miR-30a-5p is poorly expressed in drug-resistant OC cells

To find functional relevance of SOX9 regulation by miR-30a-5p, we chose four human OC cell lines A2780, SKOV3, HO-8910 and Caov3 for resistance towards DDP, and identified SKOV3 as the most resistant cell line in the panel (figure 3*a*). We then queried the expression of miR-30a-5p and SOX9 in a normal human ovarian epithelial cell line and the OC cell line panel and found miR-30a-5p to be poorly expressed, and SOX9 to be overexpressed in the OC cell lines compared to the normal human ovarian epithelial cell line. Intriguingly, we detected the lowest miR-30a-5p expression and highest SOX9 expression in SKOV3 cells, which we previously identified to be the most DDP-resistant among the ones we tested (figure 3*b*,*c*). We therefore chose SKOV3 cells for further experiments. We generated even more resistance in SKOV3 cells against DDP (SKOV3/DDP) by prolonged exposure of drug, and reassayed for miR-30a-5p expression. Intriguingly, we found an even lower expression of miR-30a-5p in SKOV3/DDP cells compared with that in SKOV3 cells (figure 3*d*), thereby highlighting a potential role of miR-30a-5p in OC chemoresistance.

**Figure 3.** miR-30a-5p is poorly expressed in DDP-resistant OC cells. (*a*) Cell inhibition rate of cell lines including A2780, SKOV3, HO-8910 and Caov3 measured by CCK-8 assay. (*b*) miR-30a-5p expression and the mRNA expression of SOX9 in a normal human ovarian epithelial cell line and four OC cell lines determined by RT-qPCR. (*c*) The protein expression of SOX9 normalized to GAPDH in a normal human ovarian epithelial cell line and four OC cell lines analysed by western blot analysis. (*d*) The expression of miR-30a-5p in drug-resistant cell line SKOV3/DDP and SKOV3 using RT-qPCR. *p < 0.05 versus IOSE 80 cells or SKOV3 cells. Measurement data were expressed as mean ± standard deviation. Comparisons among multiple groups were conducted by one-way ANOVA with Tukey's *post hoc* test. Data at different time points were compared by repeated-measures ANOVA followed by Bonferroni *post hoc* test. Cell experiment was repeated three times independently.

### 2.4. miR-30a-5p strengthens the sensitivity of OC cells to DDP

To investigate the functional effects of miR-30a-5p on OC cells, we transfected SKOV3/DDP cells with a miR-30a-5p mimic, and SKOV3 cells with a miR-30a-5p inhibitor. We then determined the expression of miR-30a-5p and SOX9 in both cell lines using RT-qPCR and western blot analyses. We found miR-30a-5p expression to be significantly increased and SOX9 expression to be decreased in SKOV3/DDP cells transfected with miR-30a-5p mimic, and miR-30a-5p expression to be profoundly diminished and SOX9 expression to be increased in SKOV3 cells transfected with miR-30a-5p inhibitor (figure 4*a*,*b*). We then used the cell counting kit-8 (CCK-8) assay as well as flow cytometric data to demonstrate that miR-30a-5p overexpression enhanced growth inhibition of SKOV3/DDP cells responding to different concentrations of DDP, decreased DDP IC_50_, induced a G1 cell cycle arrest and increased rate of apoptosis, while miR-30a-5p inhibition elicited the opposite results (figure 4*c*,*d*). In order to directly prove the role of SOX9 in this regulation, we delivered si-SOX9 into SKOV3/DDP cells and found that si-SOX9 significantly decreased DDP IC_50_, blocked cell cycle in G1 phase and enhanced the apoptosis rate significantly. Therefore, SOX9 silencing sensitized cells to DDP. In addition, we noted that the promotive effects of the miR-30a-5p inhibitor on DDP resistance could be reversed by the silencing of SOX9 (figure 4*e–g*). In summary, miR-30a-5p increases the rate of apoptosis and enhanced the sensitivity of OC cell to DDP by downregulating SOX9.

**Figure 4.** miR-30a-5p enhances the DDP sensitivity of OC cells through downregulation of SOX9. SKOV3 cells were treated with miR-30a-5p inhibitor (S + miR-30a inhibitor) or NC inhibitor (S + NC inhibitor), while SKOV3/DDP cells were treated with miR-30a-5p mimic (R + miR-30a mimic) or NC mimic (R + NC mimic). S, sensitive; R, resistant. (*a*) miR-30a-5p expression and the mRNA expression of SOX9 determined by RT-qPCR. (*b*) The protein expression of SOX9 normalized to GAPDH measured by western blot analysis. (*c*) Cell inhibition rate and DDP-IC_50_ measured by CCK-8 assay. (*d*) Cell cycle distribution and apoptosis analysed by flow cytometry. (*e*) Western blot analysis for the SOX9 protein level in response to miR-30a-5p mimic/inhibitor. (*f*) Cell inhibition rate and DDP-IC_50_ in response to si-SOX9 measured by CCK-8 assay. (*g*) Cell cycle distribution and apoptosis in response to si-SOX9 analysed by flow cytometry. *p < 0.05. Measurement data were expressed as mean ± standard deviation. Comparison between two groups was analysed by unpaired *t*-test. Data at different time points were compared by repeated-measures ANOVA, followed by Bonferroni *post hoc* test. Cell experiment was repeated three times independently.

### 2.5. Exosomes derived from SKOV3 or SKOV3/DDP cells can be delivered into OC cells

We next derived exosomes from SKOV3 cells (S-exo) and SKOV3/DDP cells (R-exo) and observed them under transmission electron microscopy (TEM) (figure 5*a*,*b*). S-exo and R-exo exosomes were both in circular membrane with a diameter of about 80–120 nm. We were able to demonstrate the expression of the specific surface markers CD63, CD9 and CD81 in both S-exo and R-exo exosomes using western blot analysis (figure 5*c*). We then incubated the OC cells with exosomes marked by PKH26. Using confocal microscopy, we demonstrated that exosomes marked by PKH26 were internalized by OC cells (figure 5*d*), which suggests that R-exo exosomes are sufficient to induce resistance to DDP in OC cells.

**Figure 5.** Exosomes derived from SKOV3 or SKOV3/DDP cells are internalized by OC cells. (*a*) Images of exosomes from SKOV3 cells (S-exo) and exosomes derived from SKOV3/DDP cells (R-exo) in 48 h culture supernatants under an electron microscope. Scale bar = 200 nm. (*b*) Size (diameter) and distribution of exosomes from SKOV3 cells (S-exo) and exosomes derived from SKOV3/DDP cells (R-exo) in culture supernatants for 48 h. (*c*) Western blot analysis of protein expression of exosome surface markers. (*d*) Confocal microscopic images of exosomes and OC cells (scale bar = 25 µm). Measurement data were expressed as mean ± standard deviation. Data between two groups were analysed by unpaired *t*-test. Cell experiment was repeated three times independently.

### 2.6. SKOV3/DDP-derived exosomal miR-30a-5p increases the sensitivity of OC cells to DDP

To study the functional mechanism of exosomes on OC cells, we analysed the function of miR-30a-5p in a co-culture system of SKOV3 cells and SKOV3/DDP cells-derived exosomes. Our results indicated that miR-30a-5p expression was significantly increased in exosomes derived from SKOV3/DDP cells transfected with miR-30a-5p mimic (figure 6*a*). Also, the expression of miR-30a-5p was significantly increased and the expression of SOX9 was progressively decreased in OC cells with overexpressed miR-30a-5p from the exosomes (figure 6*b*,*c*). By contrast, the expression of miR-30a-5p was profoundly decreased in exosomes derived from SKOV3 cells transfected with miR-30a-5p inhibitor. miR-30a-5p expression was remarkably decreased and that of SOX9 was increased in OC cells upon uptake of the exosomes. Next, using the CCK-8 assay and flow cytometry we observed that when co-cultured with exosomes derived from miR-30a-5p mimic-transfected SKOV3/DDP cells, the inhibition rate of SKOV3 cells and the apoptosis rate were increased, and DDP IC_50_ was significantly decreased, with more cells arrested in G1 phase. By contrast, SKOV3 cells co-cultured with exosomes derived from miR-30a-5p inhibitor-transfected SKOV3 cells exhibited decreased inhibition rate with higher DDP IC_50_, shorter G1 phase and a lower rate of apoptosis (figure 6*d*,*e*). Taken together the above findings suggest that miR-30a-5p derived from SKOV3/DDP-released exosomes increases the sensitivity of OC cells to DDP.

**Figure 6.** Exosomal miR-30a-5p derived from SKOV3/DDP cells enhances the DDP sensitivity of OC cells. (*a*) The expression of miR-30a-5p in exosomes determined by RT-qPCR. (*b*) The expression of miR-30a-5p and SOX9 in SKOV3 cells co-cultured with exosomes determined by RT-qPCR. (*c*) The protein expression of SOX9 normalized to GAPDH in SKOV3 cells co-cultured with exosome measured by western blot analysis. (*d*) The inhibition rate and the DDP IC_50_ measured by CCK-8 assay. (*e*) Cell cycle distribution and apoptosis analysed by flow cytometry. *p < 0.05. R + NC mimic refers to SKOV3/DDP cells transfected with NC mimic; R + miR-30a mimic refers to SKOV3/DDP cells transfected with miR-30a mimic; S + NC inhibitor refers to SKOV3 cells transfected with NC inhibitor; S + miR-30a inhibitor refers to SKOV3 cells transfected with miR-30a inhibitor; S, sensitive; R, resistant. Exosomes derived from those cells were co-cultured with SKOV3 cells. Measurement data were expressed as mean ± standard deviation. Comparison between two groups was analysed by unpaired *t*-test. Comparisons among multiple groups were conducted by one-way ANOVA with Tukey's *post hoc* test. Data at different time points were compared by repeated-measures ANOVA, followed by Bonferroni *post hoc* test. Cell experiment was repeated three times independently.

### 2.7. Exosomes carrying miR-30a-5p contribute to inhibition of tumour cell resistance by targeting SOX9

To further investigate the effect of exosomes carrying miR-30a-5p on tumour resistance *in vivo*, we subcutaneously injected nude mice with SKOV3 cells to stimulate *in vivo* tumour formation, and then injected exosomes carrying miR-30a-5p into DDP-treated tumour-bearing mice. We observed a reduction in tumour volume and weight of the nude mice after treatment with DDP. Intriguingly, both these metrics were observably reduced by injection of exosomes carrying miR-30a-5p mimic but elevated by injection of exosomes carrying miR-30a-5p inhibitor (figure 7*a*–*c*). Terminal deoxynucleotidyl transferase-mediated dUTP-biotin nick end-labelling (TUNEL)-positive apoptotic cells in the tumour tissues were notably increased by elevation of miR-30a-5p via the exosomes transfer, but reduced by injection of exosomes when miR-30a-5p was inhibited (figure 7*d*,*e*). Next, we used immunohistochemistry and western blot analysis, and found the protein expression of SOX9 in nude mice injected with exosomes carrying miR-30a-5p mimic was reduced, while that in nude mice injected with exosomes containing miR-30a-5p inhibitor was elevated (figure 7*f*). In summary, exosomes carrying miR-30a-5p restrain the expression of SOX9 and reduce tumour cell resistance *in vivo*.

**Figure 7.** Exosomes carrying miR-30a-5p inhibit tumour growth and promote apoptosis of tumour cells in nude mice. (*a*) Representative images of subcutaneous tumours in nude mice. (*b*) Tumour volume growth curves after multiple injections of exosomes. (*c*) Tumour weight after multiple injections of exosomes. (*d*) Immunohistochemical staining of SOX9 protein expression in tumours in the top; representative images of TUNEL positive cells in the bottom. Scale bar = 25 µm. (*e*) Apoptosis detected by TUNEL assay. (*f*) Protein expression of SOX9 normalized to GAPDH measured by western blot analysis. *p < 0.05 versus PBS. R + NC mimic referred to SKOV3/DDP transfected with NC mimic; R + miR-30a mimic referred to SKOV3/DDP transfected with miR-30a mimic; S + NC inhibitor referred to SKOV3 transfected with NC inhibitor; S + miR-30a inhibitor referred to SKOV3 transfected with miR-30a inhibitor; S, sensitive; R, resistant. Exosomes derived from those cells were injected into nude mice. Measurement data were expressed as mean ± standard deviation. Comparison between two groups was analysed by unpaired *t*-test. Comparisons among multiple groups were conducted by one-way ANOVA with Tukey's *post hoc* test. Data at different time points were compared by repeated-measures ANOVA, followed by Bonferroni *post hoc* test (*n* = 10).

## 3. Discussion

Rampant occurrence of drug resistance is a major challenge in OC treatment regimens [16]. A large amount of evidence has shown that circulating miRNAs carried by exosomes participate in the progression of chemoresistance in cancer cells [17]. A member of the miR-30 family, miR-30a-5p, has been implicated in the regulation of several types of cancers such as colon cancer [18], and osteosarcoma [19]. Interestingly, its role in suppressing DDP resistance has also been documented in OC [11]. Our study provides more evidence that miR-30a-5p enhances the sensitivity of the OC to DDP, and we identify this occurs through SOX9 downregulation. Using a co-culture system of exosomes and tumour cells, we demonstrate that the transfer of miR-30a-5p via exosomes from the DDP-resistant OC cells into the OC cells effectively reduces the DDP resistance (figure 8).

**Figure 8.** The proposed regulatory mechanism illustrating that exosomes carrying miR-30a-5p increased the sensitivity of OC cells to DDP by targeting SOX9. In DDP-resistant OC cells SKOV3/DDP, miR-30a-5p promoted apoptosis and inhibited cell viability by targeting SOX9 after DDP stimulation. In addition, miR-30a-5p could be transferred into exosomes from DDP-sensitive SKOV3 cells and then delivered into DDP-resistant SKOV3 cells, thereby promoting cell apoptosis, inhibiting cell proliferation and ultimately increasing chemosensitivity of DDP-resistant SKOV3 cells.

The initial motivating finding in this study was that miR-30a-5p is expressed at a lower level in drug-resistant OC cells than in drug-sensitive OC cells. From previous reports, miR-30a-5p is known to play an anti-oncogenic role in tumourigenesis. For instance, low expression of miR-30a-5p correlates with tumour metastasis, a high tumour stage, as well as tumour-capsule infiltration [20]. Additionally, induction of miR-30a-5p enhances drug sensitivity by inhibiting Beclin-1 in human small cell lung cancer [21]. miR-30a-5p is also proposed to effectively overcome the resistance of non-small cell lung cancer cells to EGFR inhibitor (Gefitinib) [22]. Likewise, a previous study has also reported that miR-30a-5p reduces the resistance of non-small cell lung cancer cells to paclitaxel [23]. Those findings are partially consistent with our observations that upregulation of miR-30a-5p contributes to sensitizing OC cells to DDP. It is generally known that exosomal miRNAs are able to control cancer cell-to-cell communication [24]. Exosomes carrying miRNAs are capable of regulating tumour resistance. For example, miR-433 released into culture media via exosomes has been shown to regulate resistance to paclitaxel in OC cells by inducing cellular senescence [25]. In a co-culture system, we further uncovered that exosomes can carry miR-30a-5p to reduce the resistance of OC cells to DDP by facilitating apoptosis. In addition, as demonstrated in a previous study that miR-30a-5p leads to inhibition of the migrating and invading capacities of OC cells [26], in this study, we further confirmed this anti-tumour effect of miR-30a-5p in ovarian tumours and further supported that the transfer of miR-30a-5p by exosomes enhances tumour cell apoptosis and reduces oncogenicity *in vivo*.

A few studies have found that miR-30a-5p exerts anti-tumour effects via targeting various oncogenes. For example, miR-30a-5p suppresses colon carcinoma development via targeting DTL [27]. In addition, miR-30a-5p suppresses prostate cancer cell growth by targeting PCLAF [28]. The present study demonstrated that miR-30a-5p targets SOX9 in OC. It has been previously reported that SOX9 is overexpressed in prostate cancer and acts as a tumour promoter gene by enhancing cell growth, angiogenesis and invasion [29]. A previous study has also identified SOX9 to be a tumour promoter in glioblastoma multiforme, and SOX9 silencing was shown to reduce temozolomide resistance of glioblastoma multiforme cells [30]. Similarly, another miRNA miR-190 increases breast cancer cell sensitivity to endocrine therapy both *in vitro* and *in vivo* through negative regulation of SOX9 [31]. Moreover, SOX9 silencing results in an enhanced sensitivity of the cervical cancer cells to DDP [31], which is partially consistent with our findings. Therefore, we consider the possibility that SOX9 might be a cancer-promoting gene in OC. Our experiments demonstrated that miR-30a-5p downregulates SOX9, which reverses DDP resistance.

In summary, we report that miR-30a-5p increases sensitivity of OC cells to DDP via targeting SOX9. Furthermore, exosomal miR-30a-5p delivered into OC cells contributes to enhanced sensitivity of OC cells to DDP *in vivo.* Thus, exosome-encapsulated miR-30a-5p might serve as a promising target to control drug resistance in OC. However, the application of this strategy may be limited by the current lack of effective exosome extraction techniques. The feasibility of such an approach is also yet to be verified in clinical trials. Future work should also be undertaken to elucidate how SOX9 controls DDP resistance in OC cells.

## 4. Material and methods

### 4.1. Microarray-based gene expression analysis

OC-associated gene expression profiles (GSE18520, GSE4122 and GSE54388) together with the annotated documents were retrieved in the Gene Expression Omnibus database (https://www.ncbi.nlm.nih.gov/geo) as shown in table 1, followed by background correction, normalization and preprocessing on expression matrix using Affy package in R language (https://www.bioconductor.org/packages/release/bioc/html/affy.html). DEGs were identified through the Limma package (http://master.bioconductor.org/packages/release/bioc/html/limma.html). DEGs were selected with log2 fold change >2.0 and adj.*p*.Val < 0.05 as a threshold. Heatmaps were plotted using pheatmap package (https://cran.r-project.org/web/packages/pheatmap/index.html). DiGSeE (http://210.107.182.61/geneSearch/) was applied to search OC-associated genes. The gene–gene interaction network was constructed after analysing the interaction between OC-associated genes and DEGs in String (https://string-db.org/). Cytoscape 3.6.0 software was used for the construction of an interaction network [32]. DIANA (http://diana.imis.athena-innovation.gr/DianaTools/index.php?r=microT_CDS/index), TargetScan (http://www.targetscan.org/vert_71/), miRDB (http://www.mirdb.org/), miRpath (http://lgmb.fmrp.usp.br/mirnapath/tools.php) and miRDIP (http://ophid.utoronto.ca/mirDIP/) were applied to predict the direct relations between miRNAs and DEGs. Venn online analysis tool (http://bioinformatics.psb.ugent.be/webtools/Venn/) was used to compare DEGs from different profiles or predicted miRNAs.

**Table 1.** OC-associated gene expression profiles.

accession	platform	organism	sample
GSE18520	GPL570	*Homo sapiens*	53 papillary serous ovarian adenocarcinomas tumour specimens and 10 normal ovarian surface epithelium
GSE4122	GPL201	*Homo sapiens*	10 normal and 32 malignant ovarian tissue
GSE54388	GPL570	*Homo sapiens*	16 serous OC tumour samples and six healthy ovarian surface epithelium samples

### 4.2. Cell culture

293T and human OC cell lines (Caov3 and SKOV3) were from American Type Culture Collection (Manassas, VA, USA). The ovarian epithelial cell line IOSE 80 and human OC cell lines (SKOV3 and HO-8910) were from BeNa Culture Collection (Beijing, China). Cells were passaged no more than six months and subjected to detection of mycoplasma and short tandem repeat. IOSE 80 cells were cultured with MCDB105/Medium 199 complete medium. OC cells were cultured in Roswell Park Memorial Institute (RPMI) 1640 medium containing 10% fetal bovine serum (FBS), 100 IU ml^−1^ penicillin and 100 µg ml^−1^ streptomycin. The 293T cells were exposed to high-glucose Dulbecco's modified Eagle's medium in an incubator at 37°C with 5% CO_2_. The cells were detached by 0.01% trypsin every 2–3 days and then conventionally passaged.

### 4.3. Dual-luciferase reporter gene assay

The target genes of miR-30a-5p were predicted on the microRNA.org website, and the relationship between miR-30a-5p and SOX9 was identified using dual-luciferase reporter gene assay. SOX9 3′-untranslated region was artificially synthesized and inserted into pGL3-control vector (Promega, Madison, WI, USA) between XhoI and BamH sites. Using site-directed mutagenesis, SOX9 mutant (SOX9-MUT) sequence was conducted on the basis of SOX9 wild-type (WT) sequence. Two recombinant plasmids named SOX9-WT, SOX9-MUT were co-transfected into HEK 293T cells (Shanghai Institute of Biological Sciences, Chinese Academy of Sciences, Shanghai, China) with miR-30a-5p mimic and the negative control (NC) of miR-30a-5p, respectively. After transfection for 48 h, the cells were lysed for determination of luciferase activity, which was measured on a Luminometer TD-20/20 (E5311; Promega, Madison, WI, USA) using a dual-Luciferase Reporter Assay System kit (Promega, Madison, WI, USA).

### 4.4. Establishment of DDP-resistant human OC cells

DDP-resistant SKOV3 cell line was induced by exposure to increasing DDP concentrations. SKOV3 cells were added to the medium containing 0.02 mg l^−1^ DDP. The dose of DDP was gradually increased until the cells were in a stable growth phase with the medium containing 0.2 mg l^−1^ DDP, which was named as SKOV3/DDP cell line. This induction culture lasted for eight months.

### 4.5. Plasmid transfection

The overexpression or inhibition of miR-30a-5p was achieved by transfection of miR-30a-5p mimic or miR-30a-5p inhibitor (Genepharma, Shanghai, China). The small interference RNA (siRNA) targeting SOX9 (si-SOX9) was used for knockdown of SOX9 (GeneCopoeia, Guangzhou, Guangdong, China). SKOV3/DDP cells were transfected with miR-30a-5p mimic, NC mimic, si-NC, si-SOX9, miR-30a-5p inhibitor in the presence of si-NC or si-SOX9, respectively. SKOV3 cells were transfected with miR-30a-5p inhibitor and NC inhibitor, respectively.

SKOV3 or SKOV3/DDP cells were seeded in a 12-well plate at a density of 1 × 10^5^ cells ml^−1^, transfected, and harvested upon growing in the logarithmic growth phase. Upon reaching 50–70% confluency, 800 µl serum-free medium was added to each well. The 12-well plate was added with the mixtures of plasmids and lipo2000 (11668027, Thermo Fisher Scientific, Waltham, MA, USA). The medium was renewed 6 h later. After transfection for 48 h, half of untreated or transfected SKOV3 and SKOV3/DDP cells were preserved. The rest were co-cultured with exosomes for the extraction of RNA and protein.

### 4.6. Exosome isolation

The exosomes were depleted from FBS by a 16 h ultracentrifugation at 1 × 10^6^ g at 4°C in a Beckman Coulter Avanti-J-25I centrifuge (Beckman Coulter, Brea, CA, USA). SKOV3 and SKOV3/DDP cells were incubated in exosome-free RPMI 1640 medium complemented with 10% FBS for 48–72 h; exosomes were extracted by an ultracentrifugation. Briefly, cell culture medium was sequentially centrifuged at 300*g* for 10 min, 2000*g* for 15 min and 12 000*g* for 30 min to remove floating cells and cellular debris, and submitted to a second ultracentrifugation in the same conditions. The 30 µl re-suspended exosome was collected in an Eppendorf tube and lysed with equal volume in radioimmunoprecipitation assay buffer. The protein concentration in exosome was determined using bicinchoninic acid (BCA) assay kit (Beyotime, Shanghai, China).

### 4.7. Transmission electron microscopy

Exosome precipitate was fixed, dehydrated, embedded and stained with uranyl acetate and lead citrate. Slices were visualized under a TEM (JEM-1010, JEOL, Tokyo, Japan). Exosomal markers were quantified by western blot analysis.

### 4.8. Co-culture

SKOV3 cells were cultured at 6-well plates with RPMI 1640 medium containing 5% FBS at a seeding density of 5 × 10^5^ cells per well. Exosome derived from SKOV3 cells (S-exo) and exosome derived from SKOV3/DDP cells (R-exo) (100 µg ml^−1^) were co-cultured with SKOV3/DDP cells for 3 days. SKOV3/DDP cells were starved for serum for 12 h before the experiment and cultured with phosphate-buffered saline (PBS) for 3 days as control.

### 4.9. Cell uptake of exosomes

The exosome of 200 pg diluted by l ml Diluent C solution was reacted with the mixture of l ml Diluent C solution and 4 µl fluorescence staining solution PKH26 for 5 min, followed by addition of 10 ml l% bovine serum albumin. The mixture was centrifuged at 100 000*g* at 4°C for 2 h so that the exosomes in the sample were enriched in the sucrose density range of 1.13–1.19 g ml^−1^. Exosomes obtained were re-suspended in complete medium. SKOV3 cells were stained with fluorescein isothiocyanate (FITC) Phalloidin (Yeasen Biotechnology Co., Shanghai, China), and the nuclei were stained with 4,6-diamidino-2-phenylindole in blue. SKOV3 cells and exosomes marked by PKH26 were co-cultured and observed under a confocal microscope.

### 4.10. CCK-8 assay

Upon reaching confluency of 80–90%, SKOV3 and SKOV3/DDP cells (2 × 10^4^ cells well^−1^) were cultured in a 96-well plate in an incubator at 37°C with 5% CO_2_ for 6–12 h. After the cell attachment, DDP in different concentrations (1, 2, 4, 8, 16 and 32 µmol l^−1^) was added to each well, and eight parallel wells were set for each DDP concentration. The control group was set by adding medium only. After 48 h, 20 µl 5 mg ml^−1^ CCK-8 solution was added for another 4-h culture. With the supernatant removal, 150 µl dimethyl sulfoxide was added into each well of the plate in a shaking table at low speed at room temperature for 10 min. Absorbance (A) at a wavelength of 490 nm was detected by an automatic microplate reader. The cell inhibition rate = 1 − (*A*_experimental group_ − *A*_control group_)/(*A*_NC group_ − *A*_control group_) × 100%. Cell growth inhibition curve was established, and 50% inhibitory concentration (IC_50_) was calculated by GraphPad Prism as cell resistance to DDP.

### 4.11. Flow cytometry

Analysis of cell apoptosis was performed using Annexin-V-FITC kit (C1065, Beyotime, Shanghai, China) according to the product specifications. Annexin-V-FITC-labelled cells were detected on a flow cytometer (BD FACSCalibur, San Diego, CA, USA).

Single cell suspensions were fixed in 1 ml 75% alcohol and stored at −20°C overnight for cell cycle analysis. The cell proportions in G0/G1, S and G2/M phases were then calculated by detecting fluorescence on the flow cytometer (BD FACSCalibur, San Diego, CA, USA).

### 4.12. Reverse transcription quantitative polymerase chain reaction

Total RNA was extracted using Trizol Reagent (Invitrogen, Carlsbad, CA, USA). Complementary DNA (cDNA) synthesis was performed using the RT-kit. The reverse transcriptase in cDNA samples was inactivated in water bath at 80°C for 5 min. The primers of miR-30a-5p, SOX9, U6 and glyceraldehyde-3-phosphate dehydrogenase (GAPDH) were synthesized by Kingsray Biotechnology Co. (Nanjing, Jiangsu, China; table 2). U6 snRNA was used as an endogenous control to normalize miR-30a-5p expression, while GAPDH was used as the endogenous control to normalize SOX9. The relative gene expression was calculated by using 2^−ΔΔCt^ method [33].

**Table 2.** Primer sequences for RT-qPCR. RT-qPCR, reverse transcription quantitative polymerase chain reaction; miR-30a-5p, MicroRNA-139-5p; SOX9, SRY-box 9; GAPDH, glyceraldehyde-3-phosphate dehydrogenase; F, forward; R, reverse.

gene	primer sequence
miR-30a-5p	F: 5′-ATTGCTGTTTGAATGAGGCTTCAGTACTTT-3′ R: 5′-TTCAGCTTTGTAAAAATGTATCAAAGAGAT-3′
SOX9	F: 5′-TTTCCAAGACACAAACATGA-3′ R: 5′-AAAGTCCAGTTTCTCGTTGA-3′
U6	F: 5′-CTCGCTTCGGCAGCACA-3′ R: 5′-AACACTTCACGAATTTGCGT-3′
GAPDH	F: 5′-GGTGAAGGTCGGTGTGAACGGATTTGG-3′ R: 5′-TGTGCCGTTGAATTTGCCGTGAGTGG-3′

### 4.13. Western blot analysis

Cells (1 × 10^6^) were lysed with lysis buffer. Supernatant was collected followed by the detection of protein concentration using BCA (PC0020, Beijing Solarbio Science and Technology Co., Ltd, Beijing, China). The isolated 50 µg proteins were separated by 10% sodium dodecyl sulphate–polyacrylamide gel electrophoresis, and then transferred to a nitrocellulose membrane (LC2005, Thermo Fisher Scientific, Waltham, MA, USA). The membrane was then blocked for 2 h with skim milk powder and probed with primary antibody of rabbit polyclonal antibodies to CD63 (ab134045), CD9 (ab223052), CD81 (ab155760), HSP70 (ab79852), SOX9 (ab185966) and GAPDH (ab181612) from (Abcam, Cambridge, UK) at 4°C overnight. The goat anti-rabbit immunoglobulin G (IgG; ab97051, Abcam, Cambridge, UK) labelled by horseradish peroxidase (HRP) served as the secondary antibody for 1 h of incubation at a room temperature. The membrane was then immersed in enhanced chemiluminescence reaction solution (BM101, Biomiga, San Diego, CA, USA) for development for 1 min in a dark room. The image was subjected to grey scale analysis using Gel-Pro Analyzer 4.0 (Media Cybernetics, Bethesda, MD, USA). The protein expression was normalized to endogenous GAPDH.

### 4.14. Tumour xenografts in nude mice

Fifty female nude mice (age four weeks, weight 14–16 g) were purchased and given subcutaneous injection of 1 × 10^6^ SKOV3 cells. Every 10 mice received injections of PBS, DDP-resistant OC cells (SKOV3/DDP cells) transfected with miR-30a mimic or NC mimic, or DDP-sensitive OC cells (SKOV3 cells) transfected with miR-30a inhibitor or NC inhibitor, respectively. When the tumour grew to 150–200 mm^3^, nude mice were administered with an intraperitoneal injection of DDP at 8 mg kg^−1^, two times a week.

The exosomes were delivered into the implanted tumours for a total of seven times, 100 µg per mouse, once every three days. Tumour maximum diameter (*L*) and minimum diameter (*W*) were measured, tumour volume was calculated as the formula: *V* = *W*^2^ × *L* × 0.52 [34], and mouse weight was measured weekly. On the 35th day, the nude mice were euthanized. The subcutaneous transplanted tumours were removed. Tumour tissues embedded with paraffin were sliced into serious at a thickness of 5 µm for other experiments.

### 4.15. Immunohistochemistry

The sections were fixed with 3% methanol H_2_O_2_ for 20 min, followed by antigen retrieval in a water bath. The tissue sections were sealed with normal goat serum (C-0005, Shanghai Haoran Biological Technology Co., Shanghai, China) for 20 min, after which the sections were incubated with rabbit antibody to β-gal (ab4761, 1 : 200; Abcam, Cambridge, UK) at 4°C overnight. Goat anti-rabbit IgG (ab6785, 1 : 1000, Abcam, Cambridge, UK) was utilized as the secondary antibody. The HRP-labelled streptavidin (0343-10000U, Imun Biotechnology Co., Beijing, China) was added for incubation at 37°C for 20 min. The sections were developed with diaminobenzidine (ST03, Guangzhou Whiga Biological Technology Co., Guangzhou, Guangdong, China), and counter-stained with hematoxylin (PT001, Shanghai Bogoo Biotechnology Co., Shanghai, China) for 1 min. After immersing in 1% ammonia water to return blue in colour, the mounted sections were observed under the microscope. Five high-power field views per slice were randomly selected with 400 cells per field of view.

### 4.16. Terminal deoxynucleotidyl transferase-mediated dUTP-biotin nick end-labelling

The cell apoptosis of tissue sections of nude mice was determined by the TUNEL kit (ml016875, Shanghai Enzyme Research, Shanghai, China). Sections were photographed under the microscope. Cells containing the brownish yellow substance or in brown yellow were determined as apoptotic cells. Five high-power fields were randomly selected from each slice with 400 cells per field chosen to count the apoptosis index (AI). AI (%) = the number of apoptotic cells/the number of total tumour cells × 100%.

### 4.17. Statistical analysis

The data were processed using SPSS 21.0 statistical software (IBM, Armonk, NY, USA). Measurement data were expressed as mean ± standard deviation. Paired data in compliance with normal distribution and homogeneity between two groups were compared by paired *t*-test, while unpaired data were analysed by unpaired *t*-test. Comparisons among multiple groups were conducted by one-way analysis of variance (ANOVA) with Tukey's *post hoc* test. Data at different time points were compared by repeated-measures ANOVA, followed by Bonferroni's *post hoc* test. A value of *p* < 0.05 was used as the threshold for statistical significance.

## Supplementary Material

Figure 2D

Reviewer comments

## Supplementary Material

Figure 3C

## Supplementary Material

Figure 4B

## Supplementary Material

Figure 4E

## Supplementary Material

Figure 5C

## Supplementary Material

Figure 6C

## Supplementary Material

Figure 7F

## Data accessibility

The datasets generated/analysed during the current study are available.
